# Intelligent Guidance and Control Methods for Missile Swarm

**DOI:** 10.1155/2022/8235148

**Published:** 2022-01-25

**Authors:** Hanqiao Huang, Xin Zhao, Xiaoyan Zhang

**Affiliations:** ^1^Unmanned System Research Institute, Northwestern Polytechnical University, Xi'an, China; ^2^Aviation Engineering School, Air Force Engineering University, Xi'an, China

## Abstract

High-speed unmanned aerial vehicles (UAVs) are more and more widely used in both military and civil fields at present, especially the missile swarm attack, and will play an irreplaceable key role in the future war as a special combat mode. This study summarizes the guidance and control methods of missile swarm attack operation. First, the traditional design ideas of the guidance and control system are introduced; then, the typical swarm attack guidance and control methods are analyzed by taking their respective characteristics into considering, and the limitations of the traditional design methods are given. On this basis, the study focuses on the advantages of intelligent integrated guidance and control design over traditional design ideas, summarizes the commonly used integrated guidance and control design methods and their applications, and explores the cooperative attack strategy of missile swarm suitable for the integrated guidance and control system. Finally, the challenges of missile swarm guidance and control are described, and the problems worthy of further research in the future are prospected. Summarizing the guidance and control methods of missile will contribute to the innovative research in this field, so as to promote the rapid development of unmanned swarm attack technology.

## 1. Introduction

High-speed unmanned aerial vehicle (UAV) is a general term for a class of aircraft used as precision-guided weapons to attack enemy targets, such as the suicide UAV, missile, and so on [1, 2]. Compared with the manned fighter, UAV has the advantages of fast dispatch speed, strong mobility, zero casualties, and convenient multi aircraft cooperative operation [3–5]. In particular, UAVs have been highly valued by military forces all over the world, with the successful application of combat UAVs, for example, “MQ-1 Predator” of the U.S. military has been applied in a variety of practical battlefields, such as Pakistan's antiterrorism, Afghanistan war, and Iraq war [6, 7]. Under the traction of hypersonic, artificial intelligence, and swarm combat technology, UAV has gradually become an important means to seize and maintain air combat advantages and will develop into a strategic and subversive force of the air force in the future [8, 9].

At present, the UAV represented by the “MQ-1 Predator” of the U.S. military needs the participation of ground controllers in all links in the attack process, using the “remote control by ground controller” combat mode. However, the attack time window is very short and the fighters are fleeting in the confrontation environment. The traditional UAV combat mode based on ground control is difficult to meet the requirements of precision attack and time-sensitive target attack. UAV autonomous attack technology has become an urgent need [10–13]. Autonomous attack is an operation mode in which UAV independently completes target data processing and fusion, situation assessment, weapon target allocation, flight control, weapon launch, attack target, and operational effectiveness evaluation in the operational airspace [14, 15]. It breaks through the limitations of “man in the loop,” makes full use of artificial intelligence technology to give full play to the operational effectiveness of UAV, and can realize the fast attack decision and control under high dynamics and strong uncertainty with multi constraints.

On the other hand, UAV is more of a combat style facing cooperative attack in actual combat applications due to the complexity of combat tasks. Compared with single UAV, multiple UAVs can form a swarm cooperative combat system with mutual cooperation, complementary advantages, and doubled efficiency in flight space. The 2009–2047 UAV system flight plan of the U.S. Air Force points out that “with the trans-swarm from automatic capability to autonomous capability, UAVs will realize multiaircraft cooperative operation, so that a single operator can monitor multiple multimission UAVs at the same time, and the attack will become more concentrated, sustained, and large-scale” [16–18]. Therefore, swarm cooperative operation will be the inevitable development trend of the multi-UAV autonomous attack operation mode.

Unmanned combat aircraft is the current cutting-edge technology and cutting-edge combat equipment, and there are only a few countries with high-performance UAVs in the world [19]. The United States has always focused on the development of unmanned combat technology. In recent years, the U.S. Department of defense has vigorously developed UAV as a subversive technology that can change the “rules of the battlefield game” and included it in the third development plan of the U.S. military “offset strategy.” As early as 1994, the U.S. military equipped the original “RQ-1 Predator” reconnaissance UAV with the laser indicator and “Hellfire” high-speed UAV to evolve into an “MQ-1 Predator” attack UAV with ground precision strike capability. By 2013, the United States successfully developed a new generation of hypersonic and stealth UAV “X–47B.” Although the project finally ran aground, however, it does not affect the progress of the U.S. military in UAV technology. In 2015, the advanced research projects agency' (DARPA) “ELF” project of the U.S. Department of defense plans to develop UAV swarm operation technology, which consists of C-130 transport aircraft shooting UAVs with mutual networking and coordination capabilities to form a “swarm” to perform attack missions. At the same time, the U.S. Air Force's concept of future operations proposes for the first time to use large airborne platforms to project multiple UAVs for cooperative attack combat tasks. In addition, the U.S. Navy is working with the Boeing team to develop small unmanned combat aircraft that can be used for cooperative antisubmarine warfare. This development project is of milestone significance for improving the U.S. military's maritime combat capability. In terms of UAV technology development, other military powers in the world are unwilling to lag behind and compete as military commanding heights one after another, for example, Israel's “Habi” suicide UAV and Europe's “neuron” UAV. According to relevant news reports in 2016, Russian military aircraft manufacturer MIG has signed an agreement with the Ministry of Trade and Industry and is preparing to implement a UAV project based on the “Ray” prototype. The internal weapon cabin of the UAV can carry 2 tons of guided weapons, including air-to-ground high-speed UAVs, gliding bombs, cruise high-speed UAV, and antiradiation high-speed UAV. The UAV project is regarded as the main support point for Russia to develop unmanned combat capability.

Although the UAV equipment developed in China initially has the ability to attack ground targets, there is still a large gap between the UAV's autonomous precision attack ability and cooperative combat ability and the United States and other countries with leading UAV autonomous combat technology, under complex conditions, especially in the high dynamic battlefield environment. The characteristics of autonomous attack of UAV swarm are that the tasks such as flight control in common airspace of multiple UAVs, perception of environment and targets, decision-making and attack trajectory planning, weapon launch, and dive attack of high-speed unmanned aerial vehicles are independently completed by UAVs and high-speed unmanned aerial vehicles, without any interference between operators and the outside world, and many cooperative factors need to be considered between UAVs and high-speed unmanned aerial vehicles in order to give full play to the advantages of swarm combat, which brings great challenges to the design of the navigation/guidance and control system of UAV and high-speed unmanned aerial vehicles. The control problem has always been the core problem of the aircraft. The error of target perception and positioning and the weakening of the performance of the cooperative control system between UAV and high-speed UAV will greatly reduce the UAV control accuracy and attack accuracy and seriously affect the precise cooperative attack efficiency of UAV. Therefore, many domestic research institutions and scholars have studied the guidance and control technology of UAV autonomous attack.

To sum up, this study summarizes and studies the swarm guidance and control of high-speed unmanned aerial vehicles in complex air combat environment. First, the separation design idea of the traditional guidance and control system is introduced, the typical swarm attack guidance and control methods are analyzed, and the limitations of traditional design methods are given. On this basis, this study focuses on the advantages of integrated guidance and control design compared with traditional design ideas, summarizes the commonly used integrated guidance and control design methods and their applications, and then explores the swarm cooperative attack strategy suitable for the integrated guidance and control system. Finally, the challenges of UAV swarm guidance and control are described, and the problems worthy of further research in the future are prospected.

## 2. Swarm Guidance and Control of the Missile

The autonomous attack diagram of unmanned combat aerial vehicle (UCAV) swarm carrying multiple missiles is shown in Figure 1. Assume that the UCAV swarm is composed of *n* UCAVs, and it performs the task of attacking *m* enemy targets. Compared with the independent attack of single UCAV, the differences of each stage of UCAV swarm independent attack are as follows:

1. UCAV aircraft swarm cooperative cruise flight segment
2. In the cruise flight phase, the swarm composed of multiple UCAVs needs to rely on a certain cooperative control mechanism to ensure the safe flight of multiple UCAVs and fly to the mission area as a whole in the form of swarm. At the same time, the cooperative factors of multiple UCAVs need to be considered in the target allocation, attack area, and optimal launch position calculation.
3. High-speed UAV dive attack section

For some key targets or special targets, a single missile is often not enough to form a complete destruction capability, and multiple missiles are required to attack the target at the same time or at a specific impact angle, respectively. Therefore, the coordination of multiple missiles is reflected in the coordinated integrated guidance and control strategy of multiple missiles in the dive attack phase. The cooperative factors among multiple missiles must be considered comprehensively in order to realize the cooperative saturation attack or angle penetration attack on specific targets.

At the end of autonomous attack, the missile guidance and control system is the key to realize autonomous and accurate attack after unmanned aerial vehicles launch missiles. The performance of the system ultimately determines the completion effect of the attack task. However, the missile guidance and control problem based on the independence of traditional guidance and control is the key to restrict the improvement of time-sensitive attack and precision attack capability of unmanned aerial vehicles and missiles in complex battlefield environment [20–22], and the intelligent control mode of integrated guidance and control can fully realize the complementary advantages between different functional models, so as to balance the differences between different external disturbances, reduce the real-time cumulative error, and improve the robustness of the overall control effectively.

### 2.1. Traditional Guidance and Control System Design Approach

As is shown in Figure 2, the traditional guidance and control system design idea of missile is to separate the guidance system from the control system and then carry out system design separately [23, 24]. The core of the traditional guidance and control design method lies in the design of guidance law. The regularly expected control command is given through the guidance law, and then, the flight control system executes the control command to control the missile to maintain a stable flight attitude and perform the task of attacking battlefield targets.

In terms of missile precision attack control, proportional guidance law was first applied to the design of the missile guidance and control system and proved to be a simple and effective method. Gu et al. [25] designed the three-dimensional proportional guidance law of missile based on the RBF neural network, which not only met the control accuracy but also improved the robustness of proportional guidance law. In 1970s, the optimal guidance law began to be widely used. Morgan et al. [26] designed the optimal guidance law with minimum energy consumption according to the specific direction constraints of the missile velocity vector.

In order to improve the killing power and operational efficiency of missiles, missile autonomous attack must meet certain impact angle constraints. At the same time, in order to carry out saturation attack on enemy targets, it is also necessary to meet time coordination and realize synchronous attack. Therefore, the research on multimissile cooperative guidance and control technology has become a hot direction. Zhang et al. [27] proposed a distributed cooperative guidance law based on offset proportional guidance based on the consistency of action time of multiple missiles and taking the action time error as feedback. This method not only handles the tracker's field of view constraints but also realizes the consistency of action time based on the fixed or variable communication network. Krizmancic et al. [28] designed the optimal guidance and control method to meet the missile terminal constraints by reasonably optimizing the allocation of acceleration commands in the guidance system based on the landing angle constraints and acceleration constraints. Tang et al. [29] first established an offset proportional guidance law for a single missile and finally formed a networked cooperative guidance and control method with landing angle and time constraints by adjusting the remaining attack time of other missiles in real time. Li and Ma [30] designed an optimal controller suitable for multimissile cooperative attack based on the idea of lead missile and slave missile. The simulation results show that this method can better meet the coordination of attack time and attack angle.

Although the traditional design has been proved to be an effective method, the time constant of the guidance loop becomes smaller and the bandwidth becomes larger at the end of missile attack, with the reduction of the relative distance between the missile and the target. At this time, the assumption of spectrum separation will no longer hold. If the traditional method is used to design the guidance system and control system, respectively, it often leads to problems such as large miss distance and flight instability. At the same time, the separation of the guidance system and control system also brings some problems, such as system design redundancy and high engineering design cost, and is not conducive to give full play to the overall potential and efficiency of weapons, which seriously restricts the precision strike capability and combat effectiveness of missiles.

## 3. Integrated Guidance and Control Approach

Integrated guidance and control (IGC), also known as guidance and control fusion, and its design idea no longer distinguish between guidance loop and control loop, but consider the two loops as a whole. The method framework is shown in Figure 3. The rudder deflection angle control command is directly generated according to the relative motion of missile target and the missile's own flight state, which can not only avoid instability but also greatly improve the guidance and control accuracy. At the same time, integrated guidance and control can also reduce the design cost of the control system, improve the overall reliability of the weapon system, promote the coordination among subsystems, and greatly improve the operational efficiency of missile [31–33]. In essence, the design of integrated guidance and control can be reduced to the nonlinear control problem of system output regulation. Because it must consider the strong coupling between the guidance and control system, it is different from the general nonlinear control method.

Since Williams et al. [34, 35] proposed the concept of IGC in 1983, scholars at home and abroad have proposed a variety of design methods for integrated guidance and control, mainly including the optimal control method, backstepping control method, sliding mode control method, trajectory linearization control method, and dynamic surface control method.

### 3.1. Optimal Control Method (OC)

Optimal control is the earliest method used for missile fusion guidance and control [36]. In fact, Williams et al. designed the IGC control system of tactical missile by using the optimal control and estimation theory in literature [34, 35], and the numerical simulation of BTT missile attacking movable target verifies the correctness of IGC concept and the effectiveness of the optimal control method. Menon and Ohlmeyer [37] transformed the IGC control problem into an optimal control problem and designed the IGC controller by using the linear quadratic regulator method. The control goal was to make the miss distance zero and ensure the stability of the missile flight state. Zhao and Zhau [38] adopted the improved exponential average method to predict the target trajectory, transformed the integrated guidance and control of the missile into a nonlinear optimization problem in finite time domain, and designed the rolling time domain IGC control strategy based on the Gaussian pseudospectrum method. Although the optimal control method is simple and effective, its deficiency lies in the lack of effective analytical solution.

### 3.2. Backstepping Control Method (BC)

As a typical nonlinear control method, backstepping control has the advantage that it can well deal with the unmatched uncertainty in the system. Therefore, it has also been applied in the design of integrated guidance and control [39, 40]. Liang et al. [41] proposed an adaptive backstepping control method for a class of IGC method design problems with input constraints. The simulation results showed that this method can not only effectively deal with the input constraints but also be robust to the system uncertainties. Cross and Shtessel [42] used the sliding mode disturbance observer technology to estimate the uncertainty of target, aerodynamic parameters, and environmental disturbance, designed the IGC backstepping control method with attack angle constraint, and proved the stability of the integrated guidance and control system based on Lyapunov theorem. The backstepping control method is based on the recursive idea from front to back. It is suitable for adaptive and robust control and has unique advantages in dealing with uncertainty. However, the repeated differential calculation of the virtual controller is too complex; in addition, this method has the problems of “item explosion” and parameter setting.

### 3.3. Sliding Mode Control Method (SMC)

When dealing with nonlinear problems, the sliding mode control method has the advantages of rapid convergence, simple algorithm, and strong robustness. At the same time, it is also the most widely used method in integrated guidance and control design [43]. Huo et al. [44] designed the integrated guidance and control system using the high-order sliding mode method. The simulation results showed that this method can not only ensure the stability of the missile system but also greatly improve the system response time and target strike accuracy. Hong et al. [45] designed an active disturbance rejection control method for missile IGC based on sliding mode control and extended state observer technology. This method can not only ensure that the missile has small miss distance and smooth flight trajectory but also make the missile robust to system uncertainty and external interference. Jian et al. [46] established a kind of reference model of missile and designed a novel control law by using the backstepping idea and sliding mode control algorithm, so that the missile can accurately attack the battlefield target with strong mobility. The biggest disadvantage of the sliding mode control method is that it has the problem of chattering. In the flight process of attacking the battlefield target, the missile not only needs to minimize the roll but also ensure its flight stability and trajectory smoothness. Therefore, the sliding mode control method has great limitations in practical application.

### 3.4. Trajectory Linearization Control Method (TLC)

As a novel and effective nonlinear tracking and decoupling control method, trajectory linearization control is more and more widely applied to the flight control system design of new missiles and UAVs because of its simple and effective control structure [47]. In terms of TLC, hypersonic vehicle is the most widely used. Shao and Wang [48] combined trajectory linearization with the active disturbance rejection control method to design an attitude tracking method for hypersonic vehicle reentry phase with bounded uncertainty. Zhu and Shen [49] proposed the IGC trajectory linearization control method for the strong coupling between various channels of hypersonic vehicle and dynamic constraints. The simulation results show that this method has great advantages over the optimal control method in control performance. Zhou et al. [50] designed a robust fusion guidance and control method for missile based on trajectory linearization control, but it only focuses on the pitch channel. Two major difficulties of the TLC method design lie in the high order of the IGC system and a large number of uncertainties in the system, which have a great impact on the control accuracy and robustness of the TLC method.

### 3.5. Dynamic Surface Control Method (DSC)

In order to overcome the problem of “item explosion” in the backstepping control method and sliding mode control method, Swaroop et al. [51] proposed the dynamic surface control method first. Its basic idea is to add a first-order low-pass filter between the design of the front and rear two-step control laws of the original backstepping control, so as to avoid the direct differentiation of some nonlinear signals in the next design. Due to the introduction of the filter, the design of each step controller is basically decoupled from the design of the previous stage. It only needs to deal with a much simpler “surface” control problem, which reduces the complexity of controller design. So far, the dynamic surface control method has been successfully applied in many engineering practices and has been applied in the design of integrated guidance and control. Li et al. [52] considered the constraints of the front view, designed a fusion guidance and control method based on barrier Lyapunov function and dynamic surface control, and proved the stability of IGC system by Barbalat lemma and Lyapunov stability theorem. Liu et al. [53] designed a dynamic surface fusion guidance and control method in the missile pitch channel for fixed targets with terminal landing angle constraints. In the cooperative fusion guidance and control, there are few literature applying the dynamic surface control method. Wang et al. [54] designed the cooperative fusion guidance and control method based on the dynamic surface control, but it is aimed at the fixed target of the pitch channel, and the variable speed in the dynamic system reduces the difficulty of IGC system design. Wang et al. [55] proposed a multimissile cooperative fusion guidance and control method based on dynamic surface control, but it is only aimed at ground fixed targets, which limits the applicability of the method to a great extent. The dynamic surface control method transforms the fusion guidance and control problem into a nonlinear regulation problem of some states of the system. The control goal is clear and the challenge is how to improve the adaptability and robustness of IGC dynamic surface control when the missile system itself has control input saturation, and there is nonlinearly parameterized nonmatching uncertainty in the system [56, 57].

In conclusion, the difference and comparison are given in Table 1.

### 3.6. Collaboration Strategy for Swarm Attack

The typical cluster cooperative attack operation diagram is shown in following two figures. The relative motion relationships of *N* missiles attacking one target in the longitudinal and lateral planes are shown in Figures 4 and 5, respectively.

When multi high-speed unmanned aerial vehicles cooperate to attack battlefield targets, they must comprehensively consider the cooperation in the flight process and meet the coordination requirements of terminal attack time or attack angle. Based on the idea of optimal control, Jeon et al. [58] proposed an attack time control guidance law for the antiship high-speed unmanned aerial vehicle. Kumar and Ghose [59] set the error term between the preset attack time and the remaining attack time, added it to the proportional guidance law, and designed a new guidance law through the sliding mode control method to ensure that the preset attack time constraints are met. Both the attack time control guidance law and the sliding mode guidance law do not fully consider the interaction and cooperation in the flight process of high-speed unmanned aerial vehicles. Therefore, references [60, 61] designed a two-layer structure of cooperative guidance framework and cooperative proportional guidance law. In the process of combat flight, the remaining attack time is shared between high-speed unmanned aerial vehicles through online data link, and adjust its own flight state in real time to achieve the coordination of the final attack time. In terms of attack angle coordination, Zhang et al. [62] designed a cooperative guidance law with attack time and attack angle constraints based on sliding mode control and comprehensively adopted line of sight rate adjustment technology and the second-order sliding mode method to meet the attack time and attack angle constraints. Jung and Kim [63] designed the offset proportional guidance law by using the backstepping control method, in which the offset term comprehensively considered the attack time error and attack angle error.

In the above research on attack time coordination, the estimation of the remaining attack time is inevitable, and its estimation accuracy has a great impact on the final guidance and control accuracy of high-speed unmanned aerial vehicle. In practical applications, it is extremely difficult to accurately estimate the remaining attack time, especially in the design of guidance law with attack time constraints, high-speed unmanned aerial vehicles often need different maneuvers to achieve the final attack time coordination. Although the cooperative guidance law proposed by Zhang et al. [64] does not need to estimate the remaining attack time, the designed controller is too special and fails when the attack lead angle is zero, so it is difficult to be used in practical engineering. In the guidance and control problem of high-speed UAV with landing angle constraints, the current research mainly focuses on the design of traditional guidance law and does not consider the limitation of hit angle of attack. Therefore, the cooperative fusion guidance and control of attack angle need to be further studied.

## 4. Challenges and Prospects

### 4.1. Challenges Faced

#### 4.1.1. The Control Accuracy and Robustness of Fusion Guidance and Control of Missile Swarm Need to be Improved

In the terminal stage of high-speed UAV attack, the traditional guidance system and control system design methods are prone to problems such as large miss distance and flight instability. In the design of integrated guidance and control, the existing integrated guidance and control methods have different degrees of shortcomings. In contrast, although the trajectory linearization control method is simple and easy to implement and has a good control effect, how to solve the high-order and large amount of uncertainty of the IGC system in this method has become two difficulties in the complex dynamic environment. The IGC control accuracy and robustness of high-speed unmanned aerial vehicle still need to be improved.

#### 4.1.2. It is Difficult to Realize the Guidance and Control Strategy of Missile Swarm

At present, only a few literatures have studied the cooperative integrated guidance and control problem, which is still in the preliminary exploration stage, and the cooperative integrated guidance and control strategy based on the estimation of remaining attack time are difficult to realize. At the same time, the existing cooperative integrated guidance and control design lacks full consideration and in-depth research on the problems of system stability and robustness caused by the nonlinearity and time variability of high-speed UAV, the perturbation of aerodynamic parameters of high-speed UAV, and the limitation of input saturation.

### 4.2. Prospect of Follow-Up Research

#### 4.2.1. Research on Parameter Tuning of IGC Controller for High-Speed Unmanned Aerial Vehicle and Missile Swarm

Most of the IGC controller parameters of high-speed UAV are obtained through certain logic derivation and repeated trial and error. Due to many control law parameters, filter constants, and disturbance observer parameters, the debugging time is long and difficult. Therefore, the research on the parameter tuning method of the cooperative IGC controller is another topic worthy of in-depth research.

#### 4.2.2. Research on Engineering Implementation of the Missile High-Speed UAV and Swarm Cooperative Control System

In the design of the control method, although some studies consider the factors such as command delay, input saturation, and dynamic limit, they do not involve the nonlinear uncertain characteristics in the actual control system, such as hysteresis and dead zone, which is still a certain distance from engineering implementation.

## 5. Conclusions

This research studies the swarm guidance and control of high-speed unmanned aerial vehicles in complex air combat environment, for example, the missile swarm. The separation design idea of the traditional guidance and control system is introduced, the typical swarm attack guidance and control methods are analyzed, and the limitations of traditional design methods are given that it seriously restricts the precision strike capability and combat effectiveness of missiles. The advantages of integrated guidance and control design compared with traditional design ideas are focused on, and the commonly used integrated guidance and control design methods and their applications are summarized. The swarm cooperative attack strategies suitable for the integrated guidance and control system are explored. Finally, the challenges of missile swarm guidance and control are described, and the problems worthy of further research in the future are prospected. The study can benefit from the future guidance and control system design, and the cooperative intelligent integrated guidance and control will be the next research hot.

## Figures and Tables

**Figure 1:** Design method of the traditional guidance and control system.

**Figure 2:** Design method of the traditional guidance and control system.

**Figure 3:** Design method of the integrated guidance and control system.

**Figure 4:** Relative motion in longitudinal plane.

**Figure 5:** Relative motion in lateral plane.

**Table 1:** The methods difference and comparison of integrated guidance and control.

Methods	Advantages	Disadvantages
Optimal control (OC)	Design is simple and easy to implement	System lacks effective analytical solution
Backstepping control (BC)	It can deal with uncertainty well	It may lead to item explosion problem
Sliding mode control (SMC)	It has rapid convergence, simple algorithm and strong robustness	It has the problem of chattering
Trajectory linearization control (TLC)	The decoupling control structure is simple	The high order and large numbers of uncertainties
Dynamic surface control (DSC)	It can overcome the item explosion problem	Robustness in input saturation needs to be enhanced

## Data Availability

The data used to support the findings of this study are included within the article.
